# Mechanistic Investigation of Curcuma Protection against Oral Submucous Fibrosis

**DOI:** 10.1155/2022/3891598

**Published:** 2022-08-09

**Authors:** Haiyan Peng, Xiaowen Jiang, Linna Cui, Yali Zhu, Zhikui Ye, Zhiming Zhang

**Affiliations:** ^1^Department of Stomatology, The First People's Hospital of Chenzhou, the First Affiliated Clinical Medical College, Xiangnan University, Chenzhou, China; ^2^Department of Oral and Maxilofacial Surgery, The Stomatology College, Southern Medical University, Guangzhou, China

## Abstract

**Objective:**

Oral submucous fibrosis (OSMF) is a chronic, fibrotic disease that affects the oral cavity, showing a high rate of malignant transformation. Curcuma exerts therapeutic potentials in many diseases including OSMF. However, the potential targets and pathways to explain the therapeutic effects of curcuma on OSMF are outside the scope of present knowledge. Herein we intend to reveal the predictive targets and potential pathways of curcuma against OSMF by a network pharmacology-based approach followed by molecular docking technology.

**Methods:**

We searched the SymMap, GeneCards, and OMIM database to obtain curcuma and OSMF common targets. The protein-protein interaction (PPI) of curcuma and OSMF common targets were then analyzed, followed by functional enrichment analysis. The best binding mode of curcuma and target proteins was analyzed by molecular docking technology.

**Results:**

We collected 290 putative targets of curcuma molecules and 600 known therapeutic targets of OSMF, with 64 curcuma and OSMF common targets sorted out. In the PPI network, there were 63 nodes with 922 edges. The node indicates protein and the line indicates PPI relation. The most enriched GO term in the BP level is “gland development”, followed by “cellular response to chemical stress”, and then “response to oxygen levels”, while the most enriched GO term in CC and MF is “membrane raft” and “cytokine receptor binding”, respectively. We also found 131 KEGG pathways significantly enriched by curcuma and OSMF common targets. The binding energy of curcuma to ALB, TNF, TP53, IL6, and VEGFA was −9.5 kcal/mol, −3.9 kcal/mol, −3.5 kcal/mol, −3.6 kcal/mol, and −8.9 kcal/mol, respectively, which suggested ALB and VEGFA were regarded as main targets involving in the potential mechanism of curcuma against OSMF.

**Conclusion:**

The present study illustrated that the therapeutic effects of curcuma on OSMF were achieved by targeting ALB and VEGFA, which giving reference to further drug design and development for OSMF.

## 1. Introduction

Oral submucous fibrosis (OSMF) is defined as a chronic scarring disease that severely affects the oral cavity, oropharynx, and sometimes the oesophagus [1, 2]. It represents a precancerous disorder and the transformation into oral squamous cell carcinoma has been found in 6%–30% cases of OSMF [1, 3]. OSMF is characterized by abnormal accumulation of collagen concomitant with progressive fibrosis in the submucosal connective tissues and limit mouth opening and tongue movement, leading to impingement on speech and swallowing [4]. OSMF is described as a multifactorial disease and mainly results from the habit of chewing betel quid and other areca nut containing products especially in Asian countries, lack of vitamin and iron, overconsumption of spicy food, and genetic susceptibility [5]. In China, men present a higher predisposition to OSF than women [6, 7]. The World Health Organization statistics, more than 5 million individuals are afflicted by OSMF worldwide, with age ranging from 8 to 80 years [8]. The mainstay of OSMF management is to minimize the annoying symptoms and increase the mouth opening to improve the quality of life of patients and further prevent malignant transformation. The current treatment strategies for OSMF mainly includes drug treatment, mouth exercise physiotherapy, and elective surgery [9]. The primary clinical drugs to treat OSMF are corticosteroids, mainly focusing on ameliorating the inflammation and reducing the collagen formation in the oral tissue [10]. Several adjuvant agents including vitamins and vasodilators, aid to relive the symptoms [11]. Mouth exercise physiotherapy alone or plus other modalities has been found to significantly increase the mouth opening [12]. Laser therapy has been introduced as a promising non-invasive technique to treat OSMF in modernized dentistry [13]. Recently, herbal derivatives or extracts have been studied by oral physicians to treat OSMF rather than commonly practiced intralesional steroids due to better patient compliance and better performance [14].

Curcumin, as a main bioactive polyphenolic compound, is extracted from the curcuma longa (also known as tumeric) that is a plant belonging to the ginger family (Zingiberaceae), originated from India, and currently grown in Southeast Asia and China [15]. Curcuma has attracted broad attention from ancient times as it owns profound biochemical and biological activities, such as antiviral, antimicrobial, anti-inflammatory, and antioxidant activities [16, 17]. Several investigations have revealed therapeutic implications of curcuma in several human diseases including diabetes [18], cancers [19], wound healing [19], rheumatic diseases [20], and ulcers [21]. Curcuma was previously studied in animal oral ulcer model, showing enhanced mucosal healing potentials [22]. Researchers treated rat models of OSMF with curcumol-loaded collage scaffold [23]. However, the potential targets and pathways to explain the therapeutic effects of curcuma on OSMF are outside the scope of present studies. Network pharmacology is burgeoning as an effective method to provide a systemic analysis of the pharmacokinetic properties of traditional Chinese medicine (TCM) by uncovering the interrelationship among drugs, targets, pathways, and disease [24]. Molecular docking is a drug design technology that simulates the geometric structure of molecules and estimates the best binding mode of small molecule drugs and its potential targets. Using both techniques in this study, we attempt to (i) construct OSMF interaction network with the targets of curcumol, (ii) decipher the mechanism elucidating the preventive role of curcuma against OSMF, and (iii) verify the potential targets of curcuma in treating OSMF.

## 2. Methods

### 2.1. Common Targets Mining

The SymMap database, accessed at http://www.symmap.org/, was retrieved to collect putative targets of curcuma. The proteins (only “*Homo sapiens*”) corresponding to the above active components were transformed into gene symbols using the UniProt database (https://www.UniProt.org/). The targets of OSMF were acquired from two public databases the GeneCards database (https://www.genecards.org/) and Online Mendelian Inheritance in Man database (OMIM, https://omim.org/). Briefly, we used “oral submucous fibrosis” as the search term to obtain disease targets (only “*Homo sapiens*”) in these two databases, with duplicates removed. The Venn diagram of the OSMF-associated targets and the putative targets of curcuma molecules was made using the R software to obtain curcuma and OSMF common targets and the corresponding network was visualized using Cytoscape software.

### 2.2. Protein-Protein Interaction (PPI) Network Construction

The curcuma and OSMF common targets were mapped into the STRING database, accessed at https://www.string-db.org/, to perform the PPI analysis. The PPI network was visualized by importing the tsv-based file to Cytoscape software (3.8.1). The species must be “*Homo sapiens*” and high confidence for interaction score must not less than 0.4. In the PPI network, nodes reflect proteins and connecting lines represent PPIs. The core genes ranked according to degree value obtained using cytoHubba plug-in of Cytoscape.

### 2.3. Functional Classification and Pathway Enrichment

Gene ontology (GO) functional analysis and pathway analysis based on the Kyoto Encyclopedia of Genes and Genomes (KEGG) were implemented to harvest the potential functions of the disease-drug common targets by using the “clusterProfiler” package in the R software. The results of GO analysis were presented at the three levels: biological processes, molecular functions, and cellular components. The GO terms at three levels and significant KEGG pathways enrichments were ranked by *P* value, and the top 20 pathways and top 10 GO functions were visualized as bar plots and bubble plots using the “Pathview” package in R software.

### 2.4. Molecular Docking Technology

Molecular docking technology is a well-recognized method to examine receptor-ligand interactions along with binding patterns and affinities. Therefore, we performed molecular docking analysis between curcuma and the top core target genes in the PPI network. The pdb format of the 3D structure of the proteins encoded by the top core target genes were downloaded from the RCSB Protein Data Bank (PDB) database, accessed at https://www.rcsb.org/. Then, we converted the pdb-based files containing curcuma and the proteins encoded by core targets into pdbqt-based files and search for active pockets. The AutoDockTools was employed to determine the binding ability of ligands and receptors. The binding energy less than 0 indicates spontaneous binding of ligand and receptor, and smaller values reflect higher binding activity.

## 3. Results

### 3.1. Identification of Curcuma and OSMF Common Targets

After searching the SymMap database, we collected 290 putative targets of curcuma molecules in total and then convert these molecule names into gene symbols in the UniProt database. With regard to the known therapeutic targets of OSMF, 600 targets were identified, with 578 collected in the GeneCards and 22 collected in the OMIM. Then, by using Venny 2.1 drawing software, we sorted 64 druggable targets of curcuma which were also therapeutic targets of OSMF (Figure 1(a)). We then used Cytoscape software to present disease-target-compound network (Figure 1(b)).

### 3.2. Key Targets in the PPI Network

We imported 64 curcuma and OSMF common targets into the STRING database for PPI analysis. As shown by the PPI network in Figure 2, there were 63 nodes with 922 edges, and those with higher degree values were regarded as corer target genes.

### 3.3. Enrichment Analysis for Curcuma and OSMF Common Targets

Next, we further analyzed 64 curcuma and OSMF common targets by GO annotation and KEGG pathway analyses. After GO analysis, 1736 GO terms, in total, were found to be significantly enriched by curcuma and OSMF common targets (*P* < 0.05).  Figure 3(a) lists the top 10 most enriched GO terms in the levels of BP, CC, and MF. The most enriched GO term in the BP level is “gland development”, followed by “cellular response to chemical stress”, and then “response to oxygen levels”, while the most enriched GO term in CC and MF is “membrane raft” and “cytokine receptor binding”, respectively. After KEGG pathway analysis, we found 131 KEGG pathways were significantly enriched by curcuma and OSMF common targets (*P* < 0.05).  Figure 3(b) lists the top 10 most enriched KEGG pathways.

### 3.4. Molecular Docking of Key Targets

The corresponding three-dimensional structures were downloaded from RCSB PDB to perform molecular docking and analysis in the AutoDockTools. ALB, TNF, TP53, IL6, and VEGFA as top 5 targets in the core PPI network were selected for molecular docking and analysis. The binding energy of curcuma to ALB, TNF, TP53, IL6, and VEGFA was −9.5 kcal/mol, −3.9 kcal/mol, −3.5 kcal/mol, −3.6 kcal/mol, and −8.9 kcal/mol, respectively. According to the principle of binding energy, a more negative docking score indicates a higher binding force between the compound and the protein. The affinity energy ≤ −5 kcal/mol is considered as high affinity, and thus ALB and VEGFA were regarded as main targets involving in the potential mechanism of curcuma against OSMF. The docking results are presented in a three-dimensional manner in Figure 4.

## 4. Discussion

Curcumin is the main component of turmeric (also known as curcuma longa), which is considered to be a non-toxic and safe substance for food uses and therapeutic purposes. Previous studies has proved its efficacy on various diseases such as type 2 diabetes mellitus [25], nonalcoholic fatty liver disease [26], and head and neck squamous cell carcinoma [27]. Although evidence indicated that Curcumin inhibited migration and metastasis of oral cancer cells [28], and turmeric oil and turmeric oleoresin exhibited antitumor activity in OSMF [29], few investigations have been done on the potential targets and pathways to clarify therapeutic value of curcuma against OSMF. Network pharmacology is a new and effective method, which changes the dogma of “one disease-one target-one drug”, and designs and analyses multi-target drug molecules to elaborate the mechanism of drug actions [30] in diseases such as diabetic nephropathy [31] and T-cell acute lymphoblastic leukemia [32]. As a silico structure-based approach, molecular docking strategies have been broadly applied to drug discovery process and identified new compounds with therapeutic significance [33].

In our study, according to network pharmacology method, we identified 64 common targets both acting on curcuma and OSMF through Venny 2.1 drawing software, and sorted the top 5 targets including ALB, TNF, TP53, IL6, and VEGFA as a result of PPI network. Human ALB gene encodes 609 amino acids and its expression is regulated by its promoter, transcription factor and intron. A case report of familial dysalbuminemic hyperthyroxinemia revealed that the patient showed extremely high serum free thyroxine concentration due to p.R242P mutation in the ALB gene [34]. Barasa et al. demonstrated that reduced serum ALB levels was found in HIV-1-infected patients following antiretroviral treatment, and this results might be attributed to rs1445776009 variants in the human ALB gene [35]. Furthermore, the role of ALB in cancers has been explored, for instance, the endometrial cancer patients with poor overall survival presented low serum ALB concentration, and ALB concentration was the independent prognostic factor for patients [36]. As reported by Bao et al. this prospective study concluded that ALB levels were negatively related to overall survival of oral cancer patients, exposing prognostic significance of ALB in oral cancer [37]. Similarly to previous study, elevated CRP/ALB ratio was observed in oral squamous cell carcinoma patients with poor overall survival [38]. TNF cytokine is a central regulator of immunity, which can promote inflammation. In the presence of pathogens, and inflammation and stress signals, TNF gene transcription is activated in a variety of cell types such as T cells, macrophages, and fibroblasts [39]. TNF-alpha located in the class III region of human leukocyte antigen belongs to TNF/TNFR cytokine family, and is involved in the malignant progression of disease. Like TNF cytokine, IL 6 type cytokine is essential for homeostasis and immunity maintenance. It is produced rapidly and instantaneously during infection and tissue injury, which promotes host defense by stimulating acute phase reaction, hematopoiesis and immune response [40]. TNF-alpha acts as a pathogenic role in the development of OSMF, a condition of precancerous lesions [41]. Increased risk of oral precancerous lesions, such as leukoplakia, oral lichen planus, and OSMF, was induced by TNF-*α* (−308) and IL-6 gene polymorphism [42]. Compared with healthy controls, the patients with oral lichen planus, oral leukoplakia, or OSMF all had elevated serum and salivary levels of TNF-*α* and IL-6 [43], and the findings were supported by another research, revealing that TNF-*α* and IL-6 levels increased in OSMF patients [44]. TP53 is a tumor suppressor gene and TP53 gene mutations, especially somatic mutation of TP53 gene, are responsible for more than 50% of human tumors [45]. TP53 mutation is considered as a potential prognostic and predictive marker along with a target of drug intervention in cancers. Varun et al. pointed out that mean labeling index of P53 for OSMF and normal mucosa was 34.6 ± 8.7 and 15.1 ± 9, respectively, indicating increased P53 was associated with malignant lesions of the oral cavity [46]. VEGFA is involved in the regulation of angiogenesis and vascular permeability. A systematic review and meta-analysis presented by Almangush et al. suggested that no direct correlation was found between VEGFA and oral tongue squamous cell carcinoma through the meta-analyses. However, VEGFA could be used as a prognostic indicator of oral tongue squamous cell carcinoma via the pooled analysis [47]. Furthermore, the patients with OSMF showed significantly higher mean serologic levels of VEGFA than that in healthy controls (*P* < 0.001) [48].

In the present study, we performed molecular docking method to evaluate the binding energy of curcuma to the top 5 targets, and ALB with -9.5 kcal/mol and VEGFA with −8.9 kcal/mol stood out. Previous studies manifested that the conjugation of curcuma and ALB increased the aqueous solubility of the drug, leading to favorable immunomodulatory activity with increase in total leukocyte count, platelet count, and viable cell count in bone marrow. Besides, this conjugation was helpful to inhibit tumor deterioration in model of mice with Dalton's lymphoma ascites [49]. Oral administration of curcumol-based supplement is a safe and effective anti-VEGF treatment in age-related macular degeneration, resulting in functional outcome improvement [50]. The results in our study revealed that ALB and VEGFA might be the main targets participating in the potential mechanism of curcuma against OSMF.

Of note, our study has several limitations. First, the findings in our study obtained by a network pharmacology-based approach followed by molecular docking technology need to be verified in cellular and animal model. Second, we need more database screening common targets to improve the reliability of analysis or gene expression profiling of OSMF sample compared to control can be used to obtain more validated targets of OSMF. Third, the expression patterns of ALB, TNF, TP53, IL6, and VEGFA, the regulation of curcuma on these targets in the setting of OSMF are warranted to receive experimental validation. Forth, the exact therapeutic mechanism of curcuma against OSMF should be clearly explained in the future, such as anti-inflammatory, antioxidant, or wound healing effects. Network pharmacology has been widely used for drug-target-pathway analysis [51], where we again emphasize the importance of this field for medical research.

## 5. Conclusion

In conclusion, the study illustrated that the therapeutic effects of curcuma on OSMF were achieved by targeting ALB and VEGFA. Accordingly, the study thoroughly elucidated the molecular mechanism responsible for the therapeutic effects of curcuma on OSMF, which not only can facilitate the design and application of curcuma but also may bring more profound therapeutics for minimize the symptoms and healing oral mucosal lesion thus improving mouth opening in the context of OSMF.

## Figures and Tables

**Figure 1:** Venny diagram of 64 curcuma and OSMF common targets (a) and disease-target-compound network (b).

**Figure 2:** PPI analysis for curcuma and OSMF common targets (a) and their degree in the PPI network (b).

**Figure 3:** The top 10 most enriched GO terms at the levels of BP, CC, and MF (a) and the top 20 most enriched KEGG pathways (b).

**Figure 4:** Molecular docking analysis of curcuma to ALB, TNF, TP53, IL6, and VEGFA.

## Data Availability

The data used to support the findings of this study are included within the article.
